This article has been retracted.

# Design and Implementation of Advanced Machine Learning Management and Its Impact on Better Healthcare Services: A Multiple Regression Analysis Approach (MRAA)

**DOI:** 10.1155/2022/2489116

**Published:** 2022-04-04

**Authors:** M. Kiruthiga Devi, Veena Prasad Vemuri, Mahalakshmi Arumugam, S. K. UmaMaheswaran, Purnendu Bikash Acharjee, Rupali Singh, Karthikeyan Kaliyaperumal

**Affiliations:** ^1^Department of Information Technology, Dr. M.G.R. Educational And Research Institute, India; ^2^NKES College at Arts, Commerce and Science, Mumbai University, India; ^3^Department of Management Studies, M S Ramaiah Institute of Technology, Bangalore 560064, India; ^4^Department of Mathematics, Sri Sairam Engineering College, Chennai, Tamil Nadu, India; ^5^Computer Science, The Assam Kaziranga University, India; ^6^Electronics and Communication Engineering, SRM Institute of Science and Technology, NCR Campus, Ghaziabad, Delhi, India; ^7^IT @ IoT-HH Campus, Ambo University, Ethiopia

## Abstract

In the current information and technology era, business enterprises are focusing in performing the process effectively by reducing the waiting time in completing the work, reduce latency and deploy the resources effectively so as to service the patient, medical practitioners, societies, and other stakeholders in an efficient manner. Hence, several organisations are using the emerging technologies so as to obtain high performance and enhance competitive edge. The advancement in machine learning, deep learning, business analytics, etc. enables the health care industry to identify the patterns based on the data collected and create a pivotal position and enhance revenues and profits in a sustainable manner. Machine learning models are considered as computational algorithms which will enable in collected the data, analyze them, and provide the necessary reports to the experts and management in order to make informed decision making. The application of advanced machine learning enables the organisation to process the image effectively, recognize the voice and enable in servicing the customers, process the available data, and identify the patterns so as to make informed decision making. The basic purpose of the study is to analyze the overall implementation of advanced machine learning approaches towards health care services for providing enhanced services, better patient engagement, and support in creating better life for them, the researchers intend to collect the closed-ended questionnaire from employees in different medical centers covering: apprehend the nature of designing and implementation of machine learning approaches in the organisation and understand the effectiveness of these tools in enhancing the sustainable growth and development of the organisation.

## 1. Introduction

The implementation of machine learning models is focused in implementing different algorithmic models which are involved in executing the specific data set and support in realising humanoid experiences so as to produce the desired results. Artificial intelligence (AI) is considered as the overall capability of the overall processor so as to accomplish the desired jobs in an effective manner.

In the current decade, companies focus in competing effectively based on analytics, the growth, and development of big data enable companies in gaining access and support in performing the analysis of large datasets. The innovations in the business analytics tend to become more desirable by the company focuses in addressing the necessity on the successful performance, and this holds more important for various forms of business operations apply them in different domains covering supply chain management, financial risk analysis, social media marketing, attracting customers, and support in managing the inventory effectively.

The main objective of implementing advanced machine learning approaches in business is to focus in understanding the business process, identify the areas to improvise, cut mundane task and thereby support in implementing better business process, deliver products and services in an effective manner, and enhance profits for all the stakeholders. [1]. The application of basic methods such as deep learning, robotics, automation, and other aspects will gradually affect the business, customers, employees, suppliers, and others. Using machine learning methods helps management to apply effective methods to collect, process, and organize data from different sources, analyze it in different ways, and develop standards and knowledge that help the organisation identify clear opportunities [2]. In addition, this information, when included in detailed toolbar links, assists management in analyzing process gray areas and designing strategies to improve operations.

It is more advantageous for the business to look at the various technologies like machine learning, deep learning, Internet of Things, and Robotics Process automation [3]. These disrupting tools support the business to achieve the desired objective in a sustainable manner, the top management by computerizing the business process enable in unleashing the potential of new technologies, use the human capital for productive and critical task rather than spending more time on routine and noncore activities. Digital competing also provides the business to perform functions with less or no human support, breakdown critical data, and can perform functions round the clock, hence, it adds value to the business at low cost [4].

The critical novelty of the study is to focus in analyzing the designing and implementation of ML approaches in enhancing health care services, and the study involves in applying the statistical tools for performing the study. The previous study was involved in using algorithms and other aspects of the ML approaches in deciphering massive volume of data; on the other hand, this study is enabled in testing using key statistical analysis. Furthermore, it also collaborates with other systems, connect through cloud and projects privacy, these features have made ML to be more unique and critical in business application and to enhance competitive position of the organisation in domestic and international markets. The critical role of artificial intelligence is shown in Figure 1 [5].

It has been regarded that the advancements in ML is now possessing strong competencies to enhance the business strategies across the business process. The emergence in such technologies boost innovation, collaborate effectively with the systems, individuals, and stakeholders so as to enhance communication. Moreover, with the advent of 5G technology, ML technologies can greatly support and collaborate with various businesses functions. The recent decade has witnessed that companies have been applying novel ML methods which address critical business functions. Moreover, ML has supported many businesses to improve cost, support in realising better productivity, reduce cost, and automate functions for realising efficiencies to support in profits.

The research gap of the study is to identify and implement better tools and techniques in order to support the application of ML models in the health care industry, it has been regarded that the health care functions are fast changing, and there is a need for offering better treatment and protocols within the specified time so as to provide better health care services. The application of ML is considered to be highly critical for business sustainability in the future and hence the executives are focusing in unleashing the potential of such technologies to add more benefits *n* each stage of customer value chain. Moreover, this study involves in applying statistical tools to test empirically the nature of ML in health care services.

This study is more focused in understanding the key determinants of advanced machine learning approaches which impacts the contemporary business organisation. The researchers are poised in understanding the major role played by ML influenced health care analytics; ML supporting in adding more value to patients, data analysis and security, optimisation of resources to enhance profits, and achieving sustainable growth in modern health care services. The ML supports not only in analyzing the data and information but also supports the health care services to analyze the areas of improvement and support in devising strategies so that all stakeholders benefit from such technologies.

## 2. Review of Literature

Wang et al. [6] have mentioned that the critical role played by ML is supporting in meeting and analyzing the large volume of data and hence organisations can support in devising critical strategies for gaining competitive edge through critical data analysis all organisation can make better decisions at quick span of time, ensuring robust competitive position. The advanced ML and other technologies also support the organisation in reducing cost, for example, the management can critically devise supply chain systems which will lower the overall transportation cost, inventory cost, etc. so that it supports in delivering the goods at faster pace.

Business organisations are now implementing machine learning and deep learning tools so that they can continuously engage with the customers, understand their requirements, and offer products and services which add more value. The ML also supports the organisation in understanding the customers better, analyze the topographical segment of the market, and deliver services to enhance the gratification.

Artificial intelligence leaves the R&D lab to enter the business world. Millions of leading industries and companies around the world combine the power of artificial intelligence and applied artificial intelligence (AAI) [7]. Most industries use nanosecond machine learning algorithms to detect fraud and improve customer satisfaction. The significant increase in the number of tools for machine learning, business platforms, and application-based tools is designed to meet business satisfaction. These advanced technologies not only condense the quality of the Internet and the software industry but also the quality of other industries such as construction, healthcare, law, vehicles, and agriculture.

Most leading companies, such as Microsoft, Facebook, Apple, Google, Amazon, Myntra, Flipkart, and IBM, fund research and development of artificial intelligence for the benefit of companies and customers. Some private functions and attributes can be predicted using artificial intelligence and machine learning algorithms from digital records of human behavior. With the help of artificial intelligence and a model for deep learning, we will be able to perform many tasks, but we will be more efficient [8]. The example of universal artificial intelligence is most visible in the form of support for speech recognition, Google, Alexa, and Siri. There are huge meetings. Almost half of Europeans, Chinese, Americans, and most Indians agree to use some form of speech recognition, and there is strong evidence that these platforms are aimed at the workplace. Brooks Brothers, WeWork, Mitsui USA, Capital One, and Vonage already use Alexa in their business model to improve business efficiency and work culture.

There is a blind spot in the progress or ownership of a state system. Innovation arises when we look at these edges. Machine learning and artificial intelligence-enabled organisms to overcome these gray areas. In medicine, it can be about analyzing the risk for the patient or launching a new analytical invention. In construction, this means predicting errors before they occur [9]. Today, it is all about technology and devices on the Internet and intranets. Companies now have the opportunity to collect more digital data, gain the insights they need, and revolutionize business and thinking. As a result, we are likely to see much-needed market development: faster markets, simpler rules and processes, dynamic transactions and transactions, higher returns, well-informed and informed customers, and motivated transactions [10]. Although the invention of most artificial intelligence creates economic development by only recognizing innovative openings and interruptions and is pleasing to the eye in modern action, a market segment that has been ignored by other business moguls or enters new markets provides connected devices [11]. Which feeds a continuous stream of data functionality, machining, manufacturing, and an automated help center on demand, robotics, and more make financial revolutions even more exciting. Because the future of the digital business revolution with artificial intelligence is intimately linked to how countries acquire their basic computerized skills in cyberspace, spacecraft, and aviation. Great attention must be paid to scalable data-driven businesses to gather more data, information, and knowledge to change the artificial intelligence environment.

## 3. Methodology

The study is confined in analyzing the key determinants of machine learning approaches in health care industry, the recent decade has witnessed an exponential growth of machine learning in modern organisation, and they are no longer focused only in collecting and storing the data, but also involved in analyzing them critically, store in a protected environment, enable in preparing critical reports, and also support in devising strategies for achieving sustainable growth and development.

The implementation of machine learning approaches enables the management in analyzing and devising different strategies in a timely manner, support in creating better products and services for adding more value to the customers, perform better analysis of the data and save them in protected environment, and also deploy the resources effectively for enhancing profits [12]. This study applies descriptive research study as the authors are focused in understanding the overall played by ML in supporting the business organisation, and the descriptive study supports in exploring deeply the concept and critically apprehend the role of the ML in companies for sustaining competition [1]. The researcher implements quantitative approach as the data were collected from both primary and secondary sources. The secondary data sources were mainly from EBSCO, and Scopus indexed journals in order to understand the previous study related to the subject area. The researchers tend to possess the descriptive research that supports the authors in creating a comprehensive understanding on the subject area and supports in performing the research more effectively.

The researcher uses questionnaire as the tool for collecting information from the sample respondents for purpose of primary data collection, the questionnaire will be closed ended and the respondents need to choose the available option presented for each question, and Likert scale is used in creating the options for questions related to critical variables. The researchers implemented nonprobability convenience sampling method so that they can choose the respondents effectively, and nearly 190 questionnaires were issued and 178 questionnaires were received from the respondents which are used for analysis.

For the purpose of data analysis IBM SPSS is used, the researchers used correlation analysis, regression analysis, and analysis of variance for testing the hypothesis.

ML influenced health care analytics

ML supporting in adding more value to patients

Data analysis and security

Optimisation of resources to enhance profits

Achieving sustainable growth in modern health care services

Hypothesis

*H*1: there is no statistical relation between ML influenced health care industry and impact on organisation to achieve sustainable growth in modern health care services.

*H*2: there is no statistical relation between ML supporting in adding more value to customers and impact on organisation to achieve sustainable growth in modern health care services.

*H*3: there is no statistical relation between data analysis and security towards impact on organisation achieve sustainable growth in modern health care services.

*H*4: there is no statistical relation between optimisation of resources to enhance profits and impact on organisation achieve sustainable growth in modern health care services.

## 4. Analysis

The data analysis is performed using IBM SPSS Package, the researchers has collected the data from respondents who are currently working in the organisation where machine learning technologies are mainly applied for various purpose, the analysis covering percentage analysis in understanding the critical influence of ML in business organisation, perform correlation analysis, regression analysis, and independent sample test of demographic variables.

From Table 1, it is noted that 37.1% of the respondents have stated that machine learning technologies support in creating effective strategic formulation and hence top management tends to use them for making quick decision and enhance their competitive edge, also, 30.9% of the respondents have strongly agreed to the statement. Whereas 16.9% were neutral to the statement, 9% have disagreed, and 6.2% have strongly disagreed to it. This has been shown graphically in Figure 2.

Based on Table 2, it is noted that 34.8% of the respondents have agreed to the statement that ML is highly critical and significant for the future, and 33.1% of the respondents have strongly agreed to the statement. It has been regarded that the top management from different organisations is now focusing in using disruptive technologies to support in decision making, engage with the customers, and deploy the resources effectively to increase revenues and profits. However, 16.3% of the respondents were neutral *t* the statement, 8.4% of them have disagreed and remaining have strongly disagreed to the statement. This is shown in Figure 3 graphically.

### 4.1. Correlation Analysis

The next analysis applied in the study is Karl Pearson's coefficient of correlation, which supports to understand the overall behavior of the independent variables and dependent variable. The value of Karl Pearson lies between -1 to +1.

From Table 3 analysis, it is noted that the coefficient of correlation between ML influenced strategy and creating sustainable growth in contemporary organisation is +0.832 and ML supporting in adding more value to customers with creating sustainable growth in contemporary organisation is +0.831. This shows that there is high positive correlation between these variables, hence, the sample respondents have mentioned that ML is one of the effective tools in supporting the organisation to formulate better strategies using data analysis, enable in adding more value to the customers by reducing the lead time in movement of goods through supply chain system, engage with the customers active, and understand their requirements effectively. Moreover, other independent variables like data analysis and security and optimisation of resources to enhance profits also possess positive association towards sustainable growth in contemporary organisation.

### 4.2. Multiple Regression Analysis

After performing correlation analyses, the researcher intends to test the best fit of the model and also analyze the impact of independent variables towards dependent variable.

Based on the output from Table 4, it is identified that *R* squared value is 0.740, hence, it can be stated that the data is best fit, furthermore, it is also noted that the major variables like ML influenced strategy; ML supporting in adding more value to customers and optimisation of resources to enhance profits has significance value of less than 0.05, hence, the alternate hypothesis is selected.

Moreover, based on the data the regression equation is formulated as Y (achieving sustainable growth in modern health care services) = 0.134 + 0.367 × ML influenced health care analytics + 0.329 × ML supporting in adding more value to patients + 0.01 × data analysis and security + 0.204 × optimisation of resources for better services in medical industry.

### 4.3. Independent Sample Test between Independent Constraints and Demographic Variables

The critical independent variables considered in the analysis are ML influenced strategy; ML supporting in adding more value to customers; data analysis and security and optimisation of resources to enhance profits. The researcher intends to perform the independent sample *T* test between demographic variables and independent constraints.

From Table 5, it can be stated that the Levene statistics positive in nature and hence null hypothesis is rejected and alternate hypothesis is accepted.

### 4.4. Overall Findings and Discussion

Based on the overall analysis, it is identified that the correlation coefficient between the variables is more than 0.700, hence, it is stated that there exist higher positive correlation between the variables, also, it is stated that the significance value of regression analysis is less than 0.05, therefore, null hypothesis is rejected and alternate hypothesis is accepted, hence, it is concluded that the variables possess statistical relation towards the business organisation to achieve sustainable growth and development.

Hence, it is noted that machine learning possesses significant support to the top management in supporting to frame strategies, deploys the resources effectively for enhancing revenues and profits, also critically analyses business process for continuous improvements so that more value can be provided to the customers.

Machine learning models are seen as computer algorithms that collect data, analyze it, and provide the reports required for experts and managers to make informed decisions [13]. By applying advanced machine learning, an organisation can efficiently process an image, recognize voice and serve customers, process available data, and recognize patterns to make informed decisions. The main purpose of applying advanced methods for machine learning in companies is to focus on understanding business processes, identifying areas for improvisation, reducing daily work, and thus improving better business processes, product, and service delivery efficient and profitable. For all concerned [14], the use of basic methods such as deep learning, robotics, automation, and more often has a gradual impact on companies, customers, employees, suppliers, and others [15]. Using machine learning methods helps management to apply effective methods to collect, process, and organize data from different sources and analyze it in different ways to create models and ideas that help the organisation identify clear opportunities.

## 5. Conclusion

It was judged that ML development already has a strong ability to improve business strategies throughout the business process. The emergence of such technologies drives innovation and works effectively with systems, individuals, and stakeholders to improve communication. The organisation's executive functions are developing rapidly, and the redesign of business processes has changed all management and executive functions. Digital transformation has forced companies to constantly innovate in order to maintain their growth and achieve their goals. Therefore, ML is crucial to the future viability of the business, and managers are focused on exploiting the potential of these technologies to provide additional benefits to each step in the value chain.

Based on the overall analysis, it can be stated that the critical factors of ML like influence on health care analytics, ML supporting in adding more value to patients, data analysis and security, and optimisation of resources for better services in medical industry possess stronger and effective influence on the health care services. Hence, it can be stated that the medical practitioners, hospitals, and radiologists can focus in using these advanced technologies for enhancing the service delivery and better patient care management.

Advanced ML and other technologies can also help an organisation reduce costs, as management can design critical supply chain systems that reduce total shipping costs, warehousing costs, and so on. Companies today use machine learning and deep learning tools to continuously interact with customers, understand their needs, and offer value-added products and services. ML also helps the organisation to better understand customers, analyze the topographic market segment, and provide services to improve satisfaction.

## Figures and Tables

**Figure 1:** Critical role of artificial intelligence.

**Figure 2:** ML supports in offering better health care services.

**Figure 3:** ML is critical for the future.

**Table 1:** ML supports in offering better health care services.

ML supports in offering better health care services	Frequency	Percent
Not at all important	11	6.2
Less important	16	9
Neutral	30	16.9
Important	66	37.1
Highly important	55	30.9
Total	178	100

**Table 2:** ML is critical for the future health care.

ML is highly critical for the future	Frequency	Percent
Not at all important	13	7.3
Less important	15	8.4
Neutral	29	16.3
Important	62	34.8
Highly important	59	33.1
Total	178	100

**Table 3:** Correlation analysis.

Karl Pearson's correlation	ML influenced health care analytics	ML supporting in adding more value to patients	Data analysis and security	Optimisation of resources for better services in medical industry	Achieving sustainable growth in modern health care services
ML influenced health care analytics	1	0.896	0.838	0.870	0.832
ML supporting in adding more value to patients	0.896	1	0.857	0.871	0.831
Data analysis and security	0.838	0.857	1	0.845	0.757
Optimisation of resources for better services in medical industry	0.870	0.871	0.845	1	0.803
Achieving sustainable growth in modern health care services	0.832	0.831	0.757	0.803	1

**Table 4:** Regression analysis.

Regression analysis	*B*	Std. error	*P* val
(Constant)	0.134	0.178	0.45
ML influenced health care analytics	0.367	0.101	0.00
ML supporting in adding more value to patients	0.329	0.098	0.00
Data analysis and security	0	0.085	0.88
Optimisation of resources for better services in medical industry	0.204	0.095	0.03
*F* value	121.342		
Sig value	0.001		
*R*	0.859a		
*R* square	0.74		

**Table 5:** Independent *T* test analysis.

Demographic variable	Independent variables	Levene's statistic	Sig value
Gender	ML influenced health care analytics	4.149	0.043
	ML supporting in adding more value to patients	10.26	0.002
	Data analysis and security	3.536	0.062
	Optimisation of resources for better services in medical industry	7.604	0.006
Age	ML influenced health care analytics	1.503	0.223
	ML supporting in adding more value to patients	0.969	0.327
	Data analysis and security	0.947	0.332
	Optimisation of resources for better services in medical industry	0.387	0.535
Type of industry	ML influenced health care analytics	0.096	0.758
	ML supporting in adding more value to patients	0.344	0.559
	Data analysis and security	0.006	0.939
	Optimisation of resources for better services in medical industry	2.572	0.111
Management cadre	ML influenced health care analytics	1.481	0.225
	ML supporting in adding more value to patients	1.15	0.285
	Data analysis and security	0.982	0.323
	Optimisation of resources for better services in medical industry	2.398	0.123
Experience	ML influenced health care analytics	0.2	0.656
	ML supporting in adding more value to patients	0.168	0.683
	Data analysis and security	0.209	0.649
	Optimisation of resources for better services in medical industry	2.112	0.149

## Data Availability

The data shall be made available on request.
